# Study on the Features of Clinical Imaging Diagnosis of Arteriosclerotic Encephalopathy

This article has been retracted.

**DOI:** 10.1155/2022/3802560

**Published:** 2022-05-04

**Authors:** Wenbo Tang, Xiaoying Du, Wei Wang, Erbo Shan, Zhonglin Nie, Chaowen Yu, Yong Gao

**Affiliations:** ^1^The First Affiliated Hospital of Jinan University, Guangzhou Guangdong 510632, China; ^2^The First Affiliated Hospital of Bengbu Medical College, Bengbu Anhui 233000, China; ^3^The Second Affiliated Hospital of Bengbu Medical College, Bengbu Anhui 233000, China

## Abstract

This paper discusses the imaging diagnostic features of arteriosclerotic encephalopathy and combines the spatial context information of local features to study the clinical imaging image copy detection algorithm. Moreover, this paper proposes a clinical imaging copy detection algorithm that combines the BOW model and spatial context embedding and a clinical imaging copy detection algorithm that combines the BOW model and global context verification. In addition, this paper applies the algorithm to the imaging diagnostic features of arteriosclerotic encephalopathy and sets up a controlled experiment to start research. The experimental research shows that the application of imaging diagnosis to the detection of subcortical arteriosclerotic encephalopathy has good clinical effects and rapid remission of patients' symptoms. The effectiveness of this method can be verified by a large number of clinical practices in follow-up studies.

## 1. Introduction

Various types of dementia are one of the diseases that seriously affect the quality of life of the elderly, and bring a heavy burden to society and families. Although there is a lot of controversy about the concept and diagnosis of subcortical arteriosclerotic encephalopathy, most scholars at home and abroad believe that it is a special type of vascular dementia. Subcortical arteriosclerotic encephalopathy is a group of diseases characterized by recurrent hypertension, stroke, and progressive dementia. Moreover, early detection, early treatment, and delaying the progression of the disease are one of the medical problems that need to be solved urgently in the 21st century [1]. The most common clinical signs of SAE are varying degrees of cognitive impairment [2].

Simultaneously, varying degrees of cognitive impairment are the primary factor affecting patients' quality of life. SAE's cognitive impairment often manifests early, although it is sneaky. When clinical discovery and diagnosis occur, the patient's cognitive impairment is often already severe [3]. The mechanism of the occurrence and development of cognitive impairment in subcortical arteriosclerotic encephalopathy is still unclear. In recent years, SAE neurobiochemical studies have shown that in addition to increased homocysteine content, changes in inflammatory cells and thyroid hormone levels are also involved in the cognitive impairment process of SAE. The neuropathological explanations of cognitive impairment in SAE are mainly biased towards white matter demyelination and damage to the neural network caused by multiple lesions. This is also one of the current opinions held by a sizable number of researchers. This shows that abnormal alterations in the architecture of the white matter may play a significant role in the onset and progression of SAE cognitive impairment. The white matter of the brain is made up of many fiber bundles that link not just different areas of the brain but also the subcortical gray matter nuclei to the cerebral cortex. It is necessary for axons to retain their normal conduction function. Once the white matter fiber bundles in the brain become pathological, it is possible for the connection of the nerve fibers associated with cognitive functions to be disrupted, resulting in varying degrees of cognitive impairment.

This paper analyzes the diagnostic features of the clinical impact of arteriosclerotic encephalopathy and analyzes its clinical imaging features to provide a theoretical reference for subsequent diagnosis and treatment of related clinical features.

## 2. Related Work

The subcortical arteriosclerotic brain was studied in the literature [4], and it was discovered that the primary pathological alterations were the obstruction of deep tiny blood veins in the white matter, which induced changes in the surrounding brain parenchyma. The basilar artery and the circle of wills harden at the same time, blood vessel thickness is uneven, and light-yellow hard plaques may be seen in the wall of the blood vessel bifurcation, leading in local vascular stenosis and even blockage, culminating in localised cerebral infarction [5].

Most people with SAE experience only typical unusual responses like headaches and dizziness in the early stages. Almost all SAE patients exhibit variable degrees of cognitive impairment as the first/only clinical symptom as the illness progresses [6]. Long-term hypertension causes hardening of tiny blood arteries in the deep brain, resulting in chronic ischemia and hypoxia in the brain tissue of SAE patients, as well as diffuse or limited demyelination. Furthermore, patients often exhibit symptoms of cerebral atrophy, which may be accompanied by a single or many luminal infarctions, scattered haemorrhages, and other pathological alterations [7]. Furthermore, the link between the deep brain white matter fibers and the cortex seems aberrant in SAE patients owing to numerous pathological abnormalities in the basal ganglia and the cerebral medulla of the semioval centre. The pathogenic process is characterized by its slow and covert nature. Reduced neurological function, cognitive dysfunction, and extrapyramidal involvement, such as Parkinson's symptoms, are all clinical manifestations. Patients may also have ataxia, sensory conduction bundle involvement, such as eccentric sensory problems [8].

The onset of SAE is slow and stealthy. Imaging signs of SAE are commonly seen before clinical symptoms, according to studies. The diagnosis of SAE patients is now based mostly on the clinical signs of growing cognitive deterioration and the performance of patients with CT and lVlRl [9]. White matter patches, bands, or extensive patches of low-density shadows in the bilateral paraventricular and semioval centre areas are common CT indications of SAE. Furthermore, the lesion's border is ambiguous, it has little space-occupying impact, and the lesion's edge is shaped like a moon, with a large diameter that is generally parallel to the lateral ventricle's body. Multiple pathological alterations, including as single or multiple luminal infarcts and scattered hemorrhagic lesions, are seen in certain SAE patients. The longer the condition is allowed to progress, the smaller the softening lesions become, and varying degrees of brain atrophy may be seen [10]. On the basis of CT images, SAE can be divided into three types according to the classification standards recommended by Gotorll. The lesions of type I patients are mainly distributed in the anterior and posterior horns of the lateral ventricle, especially the frontal lobe. Among them, the posterior part of the frontal lobe is even more important. The lesions of type II patients are scattered in the white matter of the lateral ventricle (anterior, posterior horn, and body) and the centre of the semioval, and there is no fusion between the lesions [11]. The lesions seen in type III patients merged into a film. Compared with CT, MRI has the advantages of multisequence, multidirectional imaging, clear display of anatomical structure, etc. It can clearly display the anatomical structure of the brain parenchyma, and the display of SAE lesions and the diagnosis of SAE are more accurate. MRI plain scan is mostly irregular spot patch-like abnormal signals around the lateral ventricle, T1WI is slightly low signal (higher than cerebrospinal fluid signal), and T2WI is slightly higher signal (lower than cerebrospinal fluid signal). FLAIR selects an inversion recovery sequence equal to the T1 value of free water, which attenuates the signal of free water, thereby increasing the display of bound water and the contrast intensity of abnormal tissues. In addition, most SAE lesions are often accompanied by periventricular demyelination-like changes [12]. The literature [13] demonstrates that the FLAIR sequence may increase the rate of SAE detection and overcome the volume impact and artifact interference caused by cerebrospinal fluid in standard T2WI images. Additionally, it has a superior display impact on SAE demyelinating lesions, ischemia lesions, and other types of lesions and a greater application value for enhancing SAE diagnostic accuracy. Magnetic resonance angiography (MRA) technology enables the visualization of the brain's vascular wall, shape, thickness, and occlusion.. The literature [14] showed that 3D-TOF MRA can understand the shape of the craniocerebral artery, the size of the vessel wall, and the degree of sclerosis in SAE patients. When it is combined with conventional MRI, it can indirectly reflect the pathological process of the disease, so as to obtain the involvement of perforating arteries. It has great reference value for the early diagnosis of SAE.

DWI is an imaging method for studying the microscopic motion state of water molecules. It is theoretically based on the random free diffusion of water molecules in the medium, i.e., irregular random collisions caused by temperature [15]. DWI technology is the only imaging technology that can study the motion state of water molecules in living organisms so far. It takes full advantage of MRI's sensitivity to motion detection and can reflect the microscopic state of water molecules in the human body from the molecular level. Pathological/physiological changes analyze the histological and pathological characteristics of the disease from a microscopic point of view. DWI sequence imaging is especially the most prominent for SAEs with fresh infarcts. Not only can conventional MRI and DWI identify lesions sensitively but they can also study the pathophysiological changes associated with brain parenchymal lesions, hence, increasing the diagnostic accuracy of SAE [16]. In conventional MRI sequences, the random free diffusion of water molecules in the tissue has a very small effect on the signal. We mainly use the apparent diffusion coefficient (ADC) value measured by MRI to represent the free diffusion rate of water molecules in the tissue. The ADC value can represent the average value of the diffusion of water molecules in different directions in the tissue. The more significant the free diffusion of water molecules, the greater the measured ADC value. The literature [17] examined the difference in ADC values between SAE patients and normal elderly using DWI technology. The results indicated that the ADC value (1.461-1.892) of the lesion area of SAE patients was significantly greater than that of the control group (normal elderly), indicating that there are demyelination changes and axon loss in the deep white matter lesions of SAE patients, resulting in an inability to communicate. As the speed increases, the ADC value becomes larger.

## 3. Image Feature Extraction of Clinical Images

This paper proposes a reliable and efficient global context verification mode for feature extraction of clinical images. This mode uses the global context information that matches the SIFT feature to verify and remove erroneous SIFT matching pairs, which improves the accuracy of copy detection. The detailed process of the algorithm is shown in Figure 1.

A new global context descriptor, OR-GCD, is proposed. Different from the traditional global context verification method, our global context descriptor is directly obtained from the entire image area. For each SIFT matching pair between two image pictures, we use their three attribute values, main direction, feature scale, and feature point coordinates to construct two overlapping regions based on the SIFT matching pair. After that, in each overlapping area, two types of binary vectors are obtained based on brightness and gradient, and these binary vectors are connected as the OR-GCD of the area.

To provide resistance to typical geometric assaults (such as rotation, cropping, and shearing), we create overlapping sections of pictures in order to generate robust global context descriptors. We utilize the attribute values, primary direction, and feature scale of each pair of matched SIFT features in the two image images to change the direction and scale of the two image pictures to be consistent. The overlap region between the two photos is then calculated using the coordinates of the key spots. The procedure of constructing the overlapping region is shown in Figure 2.

We assume that a pair of matched SIFT features *f*_*a*_ and *f*_*b*_ are a pair of correct matches between the original image picture A and its copy image picture B. We assume that a pair of matched SIFT features T and Y are a pair of correct matches between the original image picture A and its copy image picture B. Image B is a copy image obtained after image A undergoes three combined geometric transformation attacks: rotation, scaling, and cropping. We label the corresponding key points of the two features as *P*_*A*_ and *P*_*B*_, respectively, label their main directions as *φ*_*A*_ and *φ*_*B*_, and label their scales as *s*_*A*_ and *s*_*B*_. In figure *n*, the arrow is used to indicate the attribute value of the feature. More specifically, the position of the arrow source represents the position of the key point, and the length and direction of the arrow represent the scale and main direction of the feature, respectively.

The direction and scale of the image picture A and the image picture B can be adjusted to be consistent according to the main directions and characteristic scales of the features *f*_*a*_ and *f*_*b*_. First, the algorithm uses the feature *T* as a reference feature and rotates the image picture in the image picture A with the feature *f*_*a*_ as the origin, so that the main directions of the feature *f*_*a*_ and *f*_*b*_ are consistent. Then, the algorithm adjusts image picture A by multiplying a scale factor *s*_*B*_/*s*_*A*_ so that the scales of image picture A and image picture B are the same. If the scale *s*_*A*_ is greater than the scale *s*_*B*_, the image picture is equivalent to smoothing through a Gaussian kernel. Among them, the standard Gaussian parameter used for smoothing is set to *s*_*B*_/*s*_*A*_. The transformation process of the image picture is expressed as follows:

(1) $$\begin{array}{c} X\prime_{A}=\frac{s_{B}}{s_{A}}\left(\begin{array}{cc} \cos\left(\phi_{B}-\phi_{A}\right) & -\sin\left(\phi_{B}-\phi_{A}\right)\\ \sin\left(\phi_{B}-\phi_{A}\right) & \cos\left(\phi_{B}-\phi_{A}\right) \end{array}\right)X_{A}. \end{array}$$

Among them, *X*_*A*_ represents the coordinate of any pixel in the image picture A, and *X*′_*A*_ is the new coordinate of the point in the transformed image picture after adjustment. Through the above transformation, the direction and scale of the image picture A are adjusted to be consistent with the image picture B, as shown in Figure 2(a).

After adjusting the direction and scale of the image picture to be consistent, we need to obtain the overlapping area of the two image pictures through the coordinates of the key points. For the matching SIFT features *f*_*a*_ and *f*_*b*_ in image picture A and image picture B, we first align the coordinates of key points *P*_*A*_ and *P*_*B*_. Next, we use the following formula to calculate the overlap area:

(2) $$\begin{array}{c} R_{A}=\left\{p_{A}^{i}\in A:I\left(p_{A}^{i}\right)>0\&I\left(p_{B}^{i}\right)>0\right\}, \end{array}$$

(3) $$\begin{array}{c} R_{B}=\left\{p_{B}^{i}\in A:I\left(p_{A}^{i}\right)>0\&I\left(p_{B}^{i}\right)>0\right\}. \end{array}$$

Among them, *I*(*p*_*A*_^*i*^) and *I*(*p*_*B*_^*i*^) are the brightness of pixels *p*_*A*_^*i*^ and *p*_*B*_^*i*^, and *R*_*A*_ and *R*_*B*_ are the overlapping areas of image picture A and image picture B. Because the overlapping area is the area shared by the two images, it can still contain the same image and image content under the cropping attack.

The brightness and gradient histograms are constructed in polar coordinates, and two types of binary vectors are obtained from the two histograms: brightness-based vectors and gradient-based vectors. These two vectors will be further used to generate OR-GCD. The brightness histogram is marked as H1, which is obtained by accumulating the brightness of the pixels in each of the *M* × *N* bars. To create this histogram, we set *M* columns in the radial direction of the polar coordinate system and *N* columns in the azimuth direction. The width of each column in the radial direction and the direction angle direction are

(4) $$\begin{array}{c} {wr}_{i}=\left(\frac{\sqrt{i}-\sqrt{i-1}}{\sqrt{M}}\right)\times r, \end{array}$$

(5) $$\begin{array}{c} {wa}_{j}=\frac{2\pi }{N}. \end{array}$$

Among them, *r* is equal to half of the width of the square area, which is 200. *wr*_*i*_ and *wa*_*j*_, respectively, represent the width of the *i*-th column in the radial direction and the width of the *j*-th column in the direction angle direction. This setting can ensure that the *M* × *N* bars all have the same size, that is, *πr*^2^/*MN*. The parameters *M* and *N* are set according to specific experiments.  Figure 3(b) shows a 4 × 8 luminance histogram constructed in the polar coordinate system.

After the histogram is constructed, we use the brightness of each bar and its adjacent bars to get a vector based on the brightness. For each bar *b*_(*i*, *j*)_, its brightness is denoted as *I*_(*i*, *j*)_, and its 8 adjacent bars are denoted as (*I*_(*i*, *j*)_^1^, *I*_(*i*, *j*)_^2^, ⋯, *I*_(*i*, *j*)_^8^). For each bar on the edge of the histogram, there may be less than 8 bars adjacent to it. Therefore, this paper sets the brightness of those adjacent bars that do not exist to 0. To achieve equivalent brightness and gradient invariance to CS-LBP, we compute the brightness difference of the centrally symmetrical column and encode each brightness difference with a binary number, generating a four-dimensional binary vector indicated by *V*_(*i*, *j*)_ = (*v*_1_, v_2_, *v*_3_, *v*_4_), as shown in Figure 3(c).

(6) $$\begin{array}{c} \left\{\begin{array}{c} v_{1}=s\left(I_{\left(i,j\right)}^{5}-I_{\left(i,j\right)}^{1}\right),\\ v_{2}=s\left(I_{\left(i,j\right)}^{6}-I_{\left(i,j\right)}^{2}\right),\\ v_{3}=s\left(I_{\left(i,j\right)}^{7}-I_{\left(i,j\right)}^{3}\right),\\ v_{4}=s\left(I_{\left(i,j\right)}^{8}-I_{\left(i,j\right)}^{4}\right), \end{array}\right. \end{array}$$

(7) $$\begin{array}{c} s\left(x\right)=\left\{\begin{array}{c} 1\text{ if }x\geq 0,\\ 1\text{ if }x<0. \end{array}\right. \end{array}$$

When *M* × *N* columns generate 4-dimensional binary vectors, we connect these binary vectors to generate the final brightness-based vector, denoted as *IV* = {*Iv*_1_, *Iv*_2_, ⋯, *Iv*_*M*×*N*×4_}, and the dimension of the vector is *M* × *N* × 4.

The acquisition method of the gradient-based vector is similar to the abovementioned acquisition method of the luminance-based vector. The only difference is that we build the gradient histogram *H* by accumulating the gradient amplitude of each pixel in the column. The gradient-based vector is denoted as *GV* = {*GV*_1_, *GV*_2_, ⋯, *GV*_*M*×*N*×4_}. We connect the two vectors IV and GV to form an *M* × *N* × 8-dimensional OR-GCD, denoted as *D* = (*IV*, *GV*).

This paper compares the corresponding OR-GCD of each pair of SIFT matching features to determine whether the matching pair is true or false. In addition, the verification results of matching features between two image pictures are used to measure the similarity of the two image pictures. Thus, copy detection is realized.

We are given a pair of matching features *f*_*A*_ and *f*_*B*_, and their corresponding OR-GCD is denoted as *D*(*f*_*A*_) = (*IV*(*f*_*A*_), *GV*(*f*_*A*_)), *D*(*f*_*B*_) = (*IV*(*f*_*B*_), *GV*(*f*_*B*_)). We use the following formula to calculate their distance *Dis*(*D*(*f*_*A*_), *D*(*f*_*B*_)) and determine whether they are a pair of correct matches.

(8) $$\begin{array}{c} Dis\left(D\left(f_{A}\right),D\left(f_{B}\right)\right)=\alpha \frac{\sum_{i=1}^{M\times N\times 4}\left|{Iv}_{i}\left(f_{A}\right)-{Iv}_{i}\left(f_{B}\right)\right|}{M\times N\times 4}+\left(1-\alpha \right)\frac{\sum_{i=1}^{M\times N\times 4}\left|{Gv}_{i}\left(f_{A}\right)-{Gv}_{i}\left(f_{B}\right)\right|}{M\times N\times 4}, \end{array}$$

(9) $$\begin{array}{c} Dis\left(D\left(f_{A}\right),D\left(f_{B}\right)\right)\leq {Dis}_{TH}. \end{array}$$

Among them, *Iv*_*i*_(*f*_*A*_), *Gv*_*i*_(*f*_*A*_). *Iv*_*i*_(*f*_*B*_), and *Gv*_*i*_(*f*_*B*_), respectively, represent the *i*-th element of *Iv*(*f*_*A*_), *Gv*(*f*_*A*_), *Iv*(*f*_*B*_), and *Iv*(*f*_*B*_). *α* is a weighting coefficient, and *Dis*_*TH*_ is a preset threshold. These two parameters are determined through experiments. If *Dis*(*D*(*f*_*A*_), *D*(*f*_*B*_)) is not greater than the threshold *Dis*_*TH*_, the features *f*_*A*_ and *f*_*B*_ are considered to be a pair of correct matches. Otherwise, they are considered to be a pair of false matches and removed.

We assume that given a query image *Q* and a test image *T*, the number of correct SIFT matching pairs verified between them is *n* (*Q*, *T*), and the initial SIFT matching pair is obtained through BOW quantitative matching. The quantity is *N* (*Q*, *T*). Then, the similarity of the two images is defined as the ratio of *n* (*Q*, *T*) and *N* (*Q*, *T*), and the range of the ratio is 0-1. Then, we use the following formula to determine whether the test image *T* is a copy image of the query image *Q*, and the formula is as follows [18]:

(10) $$\begin{array}{c} \frac{n\left(Q,T\right)}{N\left(Q,T\right)}\geq {\text{Rat}}_{\text{TH}}. \end{array}$$

Among them, Rat_TH_ represents a preset threshold from 0 to 1.

We take the number of verified correct matching pairs *nr* (*QT*) in the randomly selected matching pairs and define the similarity of the image picture as *nr* (*Q*, *T*)/*NR* (0, *T*), and the similarity is the range is 0-1. We can judge whether the image picture *T* is a copy of the image picture *Q* by the following formula [19]:

(11) $$\begin{array}{c} \frac{nr\left(Q,T\right)}{Nr\left(Q,T\right)}\geq {\text{Rat}}_{\text{TH}}. \end{array}$$

Among them, Rat_TH_ represents the preset reading value from 0 to 1.

The following table summarizes the performance analysis of the quick similarity measuring approach. We can assess if two matched SIFT features are a pair of proper matches using formulas (11) and (12). We assume that the likelihood of a SIFT matching feature being validated as a proper matching feature is *p*1 for each pair of replicated image images (that is, one image picture is a copy of another image picture). We assume that the chance of a SIFT matching feature being validated as a correct matching feature is *p*2 for every pair of noncopy photos. Two conclusions may be drawn from randomly picking and validating NR SIFT matching pairs: (a) if two video pictures are copied video pictures, and the number of randomly selected matching pairs judged to be correct is denoted as *nr*_1_, then, *nr*_1_ obeys a binomial distribution, denoted as *B*_1_(*NR*, *p*_1_). The probability density function of *B*_1_(*NR*, *p*_1_) can be expressed as

(12) $$\begin{array}{c} {pdf}_{1}=\left(\begin{array}{c} NR\\ {nr}_{1} \end{array}\right)p_{1}^{{nr}_{1}}{\left(1-p_{1}\right)}^{NR-{nr}_{1}}. \end{array}$$

(b) If the two image pictures are noncopy image pictures and the number of randomly selected matching pairs judged to be correct is marked as *nr*_2_, then, *nr*_2_ also obeys a binomial distribution, marked as *B*_2_(*NR*, *p*_2_). The modulus density function of *B*_2_(*NR*, *p*_2_) can be expressed as

(13) $$\begin{array}{c} {pdf}_{2}=\left(\begin{array}{c} NR\\ {nr}_{2} \end{array}\right)p_{2}^{{nr}_{2}}{\left(1-p_{2}\right)}^{NR-{nr}_{2}}. \end{array}$$

In order to obtain *p*1 and *p*2, we selected 7500 pairs of matching features of copied images and matching features of 4 M noncopy images from the holiday data set. Then, we obtained and compared the OR-GCD corresponding to each pair of matching features to verify their correctness. Among them, the number of histogram bars *M* × *N*, the weighting parameter *α*, and the threshold value rat is set according to our specific experimental results. As a result, *p*_1_ and *p*_2_ are estimated to be 0.92 and 0.24, respectively. If we apply the proposed image similarity measurement strategy to image copy detection, we can calculate the true positive rate (TPR) Py and false positive rate (FPR) Pe according to the following formula:

(14) $$\begin{array}{c} P_{T}=\overset{NR}{\underset{NR\times {\text{Rat}}_{\text{TH}}}{\sum }}\left(\begin{array}{c} NR\\ {nr}_{1} \end{array}\right)p_{1}^{{nr}_{1}}{\left(1-p_{1}\right)}^{NR-{nr}_{1}}, \end{array}$$

(15) $$\begin{array}{c} P_{F}=\overset{NR}{\underset{NR\times {\text{Rat}}_{\text{TH}}}{\sum }}\left(\begin{array}{c} NR\\ {nr}_{2} \end{array}\right)p_{2}^{{nr}_{2}}{\left(1-p_{2}\right)}^{NR-{nr}_{2}}. \end{array}$$

Table 1 shows the calculated *P*_*T*_ and *P*_*F*_ when we use different values of NR and Rat_TH_. From Table 1, we can find that when the values of NR and Rat_TH_ are set to 15 and 0.7, we can get the most satisfactory *P*_*T*_ and *P*_*F*_, namely, 0.9950 and 0.0001. This proves that our method can theoretically obtain a higher accuracy rate only by verifying a small number of randomly selected SIFT matching pairs [20].

Therefore, we propose a fast similarity measurement strategy based on random verification. It can not only ensure that our copy detection algorithm has a high accuracy rate but also significantly improve the efficiency of copy detection.

## 4. Study on the Features of Clinical Imaging Diagnosis of Arteriosclerotic Encephalopathy

The clinical data select the treated patients with subcortical arteriosclerotic encephalopathy as the research object. Inclusion criteria: (1) patients with subcortical arteriosclerotic encephalopathy, and all patients are confirmed by pathological examination; (2) patients who can strictly follow the doctor's orders to complete the relevant examinations. Exclusion criteria: (1) patients with mental disorders; (2) patients who cannot actively cooperate with medical staff for treatment. Control group: patients are given routine testing methods, and precautions are explained to patients before testing. Observation groupImaging is used to diagnose patients based on regular tests. As an auxiliary device to CT, the inspection instrument must be stable, without radio frequency pulses, without the missile effect, and without magnetic sensitivity, and it must be difficult to get magnetized by the magnetic resonance machine and lose control [21]. Simultaneously, the therapy effects (including blood pressure, dementia status, and slurred speech scores) of the two groups of patients are documented and tallied after imaging scans. SPSS18.0 software was used to process the data; count data were tested by 2, and *n* (percentage) is used to suggest, while measurement data were tested using the *t* test; *p*0.05 shows that the difference is statistically significant. After the patients were subjected to imaging tests, it is found that the diagnosis rate of CT signs in the observation group is significantly higher than that in the control group (*p* < 0.05), as shown in Table 2.

There is no statistically significant difference between the two groups of patients through imaging examination and before and after treatment (*p* > 0.05). The treatment effects of hypertension, dementia, and slurred speech in the observation group are significantly higher than those in the control group (*p* < 0.05), see Table 3.

## 5. Conclusion

Hypertension, stroke, dementia, and neurological diseases are the most common clinical factors for imaging diagnosis of subcortical arteriosclerotic encephalopathy. Furthermore, as blood pressure rises, most hypertensive individuals experience minor headaches, dizziness, sleeplessness, and lethargy. If the remedial actions are not implemented in a timely manner, problems may develop, and symptoms such as palpitation, shortness of breath, and chest tightness will develop. When a patient experiences unconsciousness, poor breathing, numbness, and frequent physical activity, it is important to check for the development of cerebral blood clots as soon as possible. Stroke is a condition in which the function or structure of brain tissue is harmed as a result of the organisation or damage of blood arteries in the patient's brain, and it may be ischemic or hemorrhagic. In the aged, subcortical arteriosclerotic encephalopathy is a kind of vascular illness. It usually appears after the age of 50. The patient's danger steadily rises as he or she grows older. The worsening of subcortical arteriosclerosis is proportional to the severity of hypertension and arteriosclerosis in patients. Subcortical arteriosclerosis has been more common in recent years, as seen by the rise in senile illnesses. CT has the best detection effect when compared to other techniques. It works by scanning the section with precision X-ray beams, gamma rays, or ultrasonic waves, etc., converting the visible light to optical signals and then converting optical signals to electrical signals. The benefit of using imaging to monitor a patient's status is that the scanning time is short and the picture is clear. According to the findings, using imaging diagnostic to the identification of subcortical arteriosclerotic encephalopathy may increase patient detection accuracy, diagnosis outcomes for patients with subcortical arteriosclerosis, and treatment accuracy. At the same time, the application of imaging diagnosis on the other hand can enable patients with subcortical arteriosclerotic encephalopathy to receive timely and scientific treatment, which is beneficial to reduce the related complications of patients with subcortical arteriosclerotic encephalopathy, and the clinical manifestation effect is significant.

## Figures and Tables

**Figure 1:** Global context verification algorithm framework.

**Figure 2:** Construction process of overlapping area.

**Figure 3:** Standardized overlapping area and its binary vector generation.

**Table 1:** *P*_*T*_ and *P*_*F*_ calculated with different NR and Rat_TH_ values.

	0.1		0.3		0.5		0.7	
1	0.920	0.240	0.920	0.240	1	0.920	0.240	0.920
2	0.994	0.422	0.994	0.422	2	0.994	0.422	0.994
5	1	0.746	1.000	0.346	5	1	0.746	1.000
10	1	0.936	1	0.444	10	1	0.936	1
15	1	0.907	1	0.281	15	1	0.907	1

**Table 2:** Diagnostic analysis of CT signs of the two groups of patients [*n*(%)].

Group	I	II	III
Observation group	41.38%	31.04%	27.58%
Control group	45.27%	37.34%	10.34%
*X*2	3.345	4.603	6.655
*p*	<0.05	<0.05	<0.05

**Table 3:** Comparison of the effects of the two groups after imaging examination and treatment.

Group	Hypertension	Dementia	Slurred language	After care
Observation group	55.19 ± 7.35	59.72 ± 6.44	64.70 ± 5.7	63.49 ± 9.09
Control group	34.02 ± 6.44	42.12 ± 8.73	44.59 ± 4.69	40.09 ± 8.10
*t*	1.186	3.729	0.166	2.732
*p*	0	0	0	0

## Data Availability

The data used to support the findings of this study are included within the article.
